# MicroRNA-27a Suppresses the Toxic Action of Mepivacaine on Breast Cancer Cells via Inositol-Requiring Enzyme 1-TNF Receptor-Associated Factor 2

**DOI:** 10.1155/2023/1153034

**Published:** 2023-04-10

**Authors:** WenHong Fu, XiaoLing Hu, GengZhang Li, SongTao Liu

**Affiliations:** ^1^Department of Anesthesiology, Nanhua Hospital Affiliated to Nanhua University, ShaoYang 422001, Hunan Province, China; ^2^Department of Anesthesiology, The First Affiliated Hospital of University of South China, Hengyang City 421000, Hunan Province, China

## Abstract

**Objective:**

To investigate the toxic effects of microRNA-27a on breast cancer cells through inositol-acquiring enzyme 1-TNF receptor-associated factor 2 inhibition by mepivacaine.

**Methods:**

The elevation of miR-27a in MCF-7 of BCC lines was measured, and groups were set up as control, mepivacaine, and elevated groups. Cells from each group were examined for inflammatory progression.

**Results:**

Elevated miR-27a in MCF-7 cells was able to distinctly augment the cell advancement (*P* < 0.01) and decline cell progression (*P* < 0.01). Meanwhile, miR-27a reduced the content of intracellular inflammatory factors IL-1*β* (*P* < 0.01) and IL-6 (*P* < 0.01), elevated the content of IL-10 (*P* < 0.01), suppressed levels of cleaved-caspase-3 and p-signal transducer and activator of transcription-3 (STAT3) (*P* < 0.01), and increased Bcl-2/Bax (*P* < 0.01).

**Conclusion:**

Elevated miR-27a in MCF-7 of BCC lineage was effective in reducing the toxic effects of mepivacaine on cells and enhancing cell progression. This mechanism is thought to be related to the activation of the IRE1-TRAF2 signaling pathway in BCC. The findings may provide a theoretical basis for targeted treatment of BC in clinical practice.

## 1. Introduction

Breast cancer (BC) is a malignant tumor that has a critical impact on the healthy lives of women worldwide, with high morbidity and mortality rates, and the number of BC patients worldwide is increasing year-by-year [1]. With the continuous progress in clinical medicine and health screening, the mortality rate of BC has been effectively controlled, and currently, methods including surgical resection, chemotherapy, and radiotherapy are continuously used to cure BC patients [2]. However, the pathogenesis of BC and the factors affecting the prognosis of BC patients are still unclear. MicroRNA (miR)-27a is a tumor-promoting factor, and in addition, abundant evidence suggests that miR-27a is elevated in tumor cells of cervical cancer, kidney cancer, and BC patients; meanwhile, miR-27a can effectively accelerate the transformation of epithelial cells to mesenchymal cells and expand tumor cell invasion and metastasis [3]. The literature [4] declared that miR-27a was significantly elevated in BC tissues compared to paraneoplastic tissues and almost correlated with the malignancy of tumors. In BC patients with low tumor pattern-metastasis (TNM) stage, miR-27a was significantly decreased compared to patients with high TNM stage.

Inositol-acquiring enzyme 1-TNF receptor-associated factor 2 (IRE1-TRAF2) is an important signaling pathway for maintaining endoplasmic reticulum homeostasis [5]. The literature [6] showed that the inhibited inositol-requiring enzyme 1-TNF receptor-associated factor 2 (IRE1-TRAF2) signaling pathway can effectively inhibit the proliferation of BCC. The literature [7] clearly indicated by immunofluorescence that IRE1-TRAF2 was significantly elevated in BC tissues compared to paraneoplastic tissues. Mepivacaine, as a new type of medium-acting local anesthetic drug used in clinical anesthesia, has a long half-life, rapid onset, and high potency, and its anesthetic effect is superior to other local anesthetics [8]. The literature [9] clarified that mepivacaine significantly inhibits the proliferation of gastric cancer (GC) cells and reduces tumor volume in GC patients, and the mechanism is supposed to be almost related to the activation of inflammatory response and stimulation of inflammatory factor release in GC cells. Activation of the inflammatory response can modulate the biological characteristics of a wide range of tumors [10]. However, the effect of mepivacaine on BCC progression is unknown, and the effect of miR-27a on the cytotoxicity of mepivacaine on BC and on the regulation of ITRE-TRAF2 is unclear.

This project intended to assess the impact of miR-27a on the cytotoxicity of mepivacaine on BCC via in vitro experiments, and whether it exerted a part via modulating the IRE1-TRAF2 signaling pathway was further analyzed to offer a theoretical basis for clinical treatment of BC patients.

## 2. Materials and Methods

### 2.1. Materials and Instruments

Human BC cell line MCF-7 (Cell Resource Center, SIBS, CAS, Kunming, China), 3-(4,5-dimethylthiazol-2-yl)-2,5-diphenyltetrazolium bromide (MTT) reagent (Sigma, USA), Dulbecco's Modified Eagle Medium (Heclone, USA), Hoechst33258 kit, interleukin (IL)-1*β* kit, IL-6 kit, and IL-10 kit (BOSTER Biological Technology Co. Ltd., Wuhan, Hubei, China), the terminal transferase uridyl nick end labeling staining kit (Beyotime Institute of Biotechnology, Shanghai, China), SYBR Premix Ex Taq kit, Prime Script RT reagent Kit (Takara Bio Inc., Otsu, Shiga, Japan), Rabbit- Bcl-2, Rabbit-Bax, Rabbit-cleaved-caspase-3, Rabbit-p-STAT3, Rabbit-STAT3, Rabbit-IRE1, Rabbit-TRAF2 and Rabbit-glyceraldehyde-3-phosphate dehydrogenase (GAPDH) (Cell Signaling Technologies (CST), Beverly, MA, USA), cell culture dishes (Heclone, USA), microplate readers (Omega Bio-Tek Inc., Norcross, GA, USA), qPCR instruments (Germany Illumina-Eco, Germany), thermostat water bath (Shanghai Yiheng Technology Co., Ltd., Shanghai, China), cell incubators (ThermoFisher Scientific, Waltham, MA, USA), fluorescence microscope (Nikon corporation, Japan), and pipettor (Eppendorf AG, Germany). Other reagents whose source is not indicated are identified in the assay.

### 2.2. Construction of Elevated miR-27a Cell Line

Plasmids were treated with 1-25(OH)2D for 48 hr. Cells were transfected with Lipofectamine 3000, strictly according to the instructions of the transfection reagent. Blank plasmids were used as controls, divided into blank control, negative control (transfected blank plasmids), and miR-27a (transient enhancement of miR-27a in MCF-7 cells). With the cell density adjusted to 1 × 10^5^ cells/mL, cells were seeded in 12-well plates, and the serum-free medium was replaced after culture for 24 hr. The mixture of the elevated miR-27a and the vacant plasmids was with Lipofectamine 3000, separately, gentle oscillation and blending were conducted, and incubation was at room temperature for 5 min. The addition of 100 *μ*L of mixed liquor was to each cell orifice, incubation was in an incubator for 36 hr, and collection of the cells in each group was to examine miR-27a in the cells.

### 2.3. Test the Grouping of miR-27a in the Cells via qPCR

The culture of collection of the successfully transfected cells was unceasingly in an incubator. Trizol reagent was added to each group of the cells, total RNA of each group was extracted, and the purity and concentration of RNA in each group were determined. Total RNA as a template was to be reversely transcribed into complementary DNA (cDNA). The design of qPCR primers was via Primer 6.0 in line with the sequence of the target gene in GenBank. The adoption of GAPDH was as an internal reference. The primers were synthesized (all Synbio Tech, Jiangsu, China). As shown in Table 1 exertion of 2^−*ΔΔ*Ct^ was to calculate the relative expression of genes in each group of the cells and adoption of miR-27a/GAPDH was to denote miR-27a in each group. The transfected cells were collected for culture and set as the elevated (addition of 3 *μ*g mepivacaine), and exertion of the untransfected MCF-7 cells was as the control and the mepivacaine (addition of 3 *μ*g mepivacaine).

### 2.4. The Impact of miR-27a on the Cell Proliferation

The adjustment of the cell density of each group was to 1 × 10^4^ cells/mL, seeding was in 96-well plates, and culture was separately in a constant temperature incubator for 12 hr. Three micrograms mepivacaine was added in the cells of the mepivacaine in a constant temperature incubator for 24, 48, and 72 hr. After the drug treatment, the culture of addition of a moderate amount of MTT was respectively for 4 hr. Appropriate amount of dimethyl sulfoxide was added and shaked for 10 min for mixing. The parameters of the multifunctional microplate reader were adjusted to 450 nm wavelength. In addition, the optical density of each group was measured and cell proliferation was calculated.

### 2.5. The Influence of miR-27a on the Cell Apoptosis

The adjustment of the cell density was to 1 × 10^5^ cells/mL, seeding was in 6-well plates, and culture of accretion of a right amount of complete medium was in a constant temperature incubator for 12 hr. Meanwhile, the culture of accretion of 3 *μ*g mepivacaine in the cells of the mepivacaine was performed. Accretion of a right amount of 4% paraformaldehyde was to fix the cells and incubation of addition of moderate amount of Hoechst 33258 stain was conducted. The record of the apoptosis of each group was with a fluorescence microscope. The dark blue ones were the normal cells and the bright blue nuclei were the apoptotic cells.

### 2.6. The Impact of miR-27a on the Cell Migration

The adjustment of the cell density was to 1 × 10^5^ cells/mL, seeding was in six-well plates, and culture of addition of a right amount of complete medium was in a constant temperature incubator for 12 hr. The culture of accretion of 3 *μ*g mepivacaine in the cells of the mepivacaine was exerted. The adoption of a pipette spear tip was to make a moderate-sized scratch on the culture plate. The culture of accretion of a moderate amount of culture medium was performed. The observation of the cell growth under a microscope and assessment of the migration capacity of each group were exerted.

### 2.7. The Influence of miR-27a on the Cell Inflammatory Factors

The adjustment of the cell density was to 1 × 10^5^ cells/mL, seeding was in six-well plates, and culture of addition of complete medium was performed for 12 hr. The culture of accretion of 3 *μ*g mepivacaine in the cells of the mepivacaine was conducted for 48 hr, discard of the supernatant was conducted, and collection of the cells in each group was as a standby. The enzyme-linked immunosorbent assay kits for IL-1*β*, IL-6, and IL-10 were used to detect the levels of inflammatory factors in each group, and the parameters of the multifunctional microplate reader were adjusted to 450 nm wavelength. In addition, the absorbance values of each group were measured and the contents of IL-1*β*, IL-6, and IL-10 in each group were calculated.

### 2.8. The Influence of miR-27a on Apoptosis-Correlated Proteins and IRE1-TRAF2 Signaling Pathway

The adjustment of the cell density was to 1 × 10^5^ cells/mL, seeding was in 6-well plates, and culture of addition of complete medium was performed. The culture of accretion of 3 *μ*g mepivacaine in the cells of the mepivacaine was exerted, discard of the supernatant was conducted, and collection of the cells in each group was as a standby. An appropriate amount of radioimmunoprecipitation assay lysis buffer was added to the cell suspension and tumor tissue of nude mice to extract the total protein. The protein concentration of each group was determined using the bicinchoninic acid protein quantification kit, and the protein was heated with the loading buffer. Then, sodium dodecyl sulfonate gel was used to separate the protein, and the treated protein was transferred to a polyvinylidene fluoride membrane via wet membrane transfer method and blocked with fresh 5% skim milk powder. Different protein bands was cut in line with the molecular weight of the protein. The incubation of Rabbit-Bcl-2, Rabbit-Bax, Rabbit-cleaved-caspase-3, Rabbit-p-signal transducer and activator of transcription-3 (STAT3), Rabbit-STAT3, Rabbit-IRE1, Rabbit-TRAF2, and Rabbit-GAPDH was performed, separately. The incubation of the corresponding secondary antibody conjugating with horseradish peroxidase at the temperature for 1 hr was conducted. Protein bands was placed to develop on a developing machine, and calculation of the corresponding proteins in each group was via cleaved-caspase-3/GAPDH, p-STAT3/STAT3, Bcl-2/Bax, IRE1/GAPDH, and TRAF2/GAPDH.

### 2.9. Statistical Analysis

The manifestation of the study results was as mean ± standard deviation (SD). In this study, SPSS 22.0 software was used to analyze the data. Exertion of each group of the data was via one-way analysis of variance (ANOVA). After the homogeneity of variance test, the pairwise comparison was via the Bonferronic method if the variance was homogeneous, while the Welch method was adopted if the variance was not homogeneous. *P* < 0.05 was accepted as indicative of distinct differences.

## 3. Results

### 3.1. Construction of Elevated miR-27a Cell Line

Test of miR-27a in the cells of each group was exerted, as shown in Figure 1. miR-27a expression in the cells of the miR-27a group was elevated compared to the blank group and the negative control group (*P* < 0.01).

### 3.2. miR-27a Is Available to Repress the Impact of Mepivacaine on BCC Proliferation

The effect of miR-27a on the proliferation of BCC MCF-7 was tested, as shown in Figure 2. MTT assay of cell proliferation in each group, the treatment of cell proliferation was with mepivacaine for different times, as shown in Figure 2(a), the treatment of cell proliferation after 48 hr was with mepivacaine, as shown in Figure 2(b). The proliferative capacity of mepivacaine was severely reduced compared to the control group (*P* < 0.01), while the elevated proliferative capacity significantly exceeded that of mepivacaine (*P* < 0.01).

### 3.3. miR-27a Is Available to Repress the Influence of Mepivacaine on BCC Apoptosis

The effect of elevated miR-27a on apoptosis of BCC MCF-7 cells was examined by Hoechst 33,258 staining, as shown in Figure 3. Figures 3(a) and 3(b) are micrographs and statistical plots, respectively. Compared with the cells in the control group, apoptosis was sharply enhanced in mepivacaine group (*P* < 0.01), and apoptosis in elevated cells was sharply decreased compared with mepivacaine group (*P* < 0.01).

### 3.4. miR-27a Is Able to Restrain the Impact of Mepivacaine on BCC Migration

The effect of miR-27a on the migratory capacity of BCC MCF-7 was investigated, as shown in Figure 4, with micrographs and statistical plots in Figures 4(a) and 4(b), respectively. The cell migratory capacity was severely decreased with mepivacaine compared with the control (*P* < 0.01), whereas the elevated cell migratory capacity was significantly enhanced with mepivacaine (*P* < 0.01).

### 3.5. miR-27a Is Able to Suppress the Influence of Mepivacaine on Inflammatory Factors in BCC

The effect of miR-27a on the content of inflammatory factors in BCC MCF-7 was assessed, as shown in Figure 5, with the contents of IL-1, IL-6, and IL-10 in Figure 5(a)–5(c), respectively. Compared with the control group, the contents of IL-1 and IL-6 were severely increased in mepivacaine (*P* < 0.01) and sharply decreased in IL-10 (*P* < 0.01); the contents of IL-1 and IL-6 were significantly decreased in the elevated cells compared with mepivacaine (*P* < 0.01), while the contents of IL-10 were sharply increased compared with mepivacaine (*P* < 0.01).

### 3.6. miR-27a Is Available to Suppress the Influence of Mepivacaine on Apoptosis-Correlated Proteins in BCC

The effect of miR-27a on apoptosis-related proteins in BCC MCF-7 was assessed as shown in Figure 6, with protein band plots and Bcl-2/Bax statistics in Figures 6(a) and 6(c), respectively, and cleaved-caspase-3 and p-STAT3 proteins in Figures 6(b) and 6(d), respectively. Intracellular cleaved-caspase-3 and p-STAT3 were enhanced in mepiquat compared to control (*P* < 0.01) and Bcl-2/Bax was severely decreased (*P* < 0.01); elevated intracellular cleaved-caspase-3 and p-STAT3 were sharply decreased relative to mepiquat (*P* < 0.01) and Bcl-2/Bax was severely enhanced relative to mepivacaine (*P* < 0.01).

## 4. Discussion

Epidemiological studies have shown that BC ranks first among new tumors in women and is a significant contributor to female mortality [11]. In addition, the clinical management of BC remains pessimistic. Mepivacaine is a commonly used clinical anesthetic that is constantly used as a substitute for lidocaine in a variety of procedures [12]. Mepivacaine acts as an anesthetic agent by stabilizing the cell membrane of neurons and effectively blocking the conduction of nerve impulses. The literature [13] declared that mepivacaine is toxic to tumor cells and that appropriate concentrations of mepivacaine are capable of causing apoptosis of tumor cells. Clinical evidence from the past few years also clarifies that the toxic effect of mepivacaine on tumor cells is also almost related to the type of tumor [14].

A large body of evidence suggest that miRNAs are involved in multiple processes of diverse tumorigenesis and development and tumor cell apoptosis, and the relevance of abnormal miRNAs is associated with the formation of almost all kinds of tumors [15]. Elevated miR-27a in multiple tumor cells regulates the progression of tumor cells. The literature [16] indicated that miR-27a was significantly enhanced in tumor tissues of patients with hepatocellular carcinoma (HCC) with lymph node metastases compared to those without metastases. The literature [17] thoroughly explored the effect of miR-27a on the toxic effects of mepivacaine on BCC MCF-7 by constructing cell lines with elevated miR-27a in vitro. The literature [18] showed that elevated miR-27a could effectively inhibit the toxic effects of mepivacaine on MCF-7 cells. The literature [19] clearly indicated that the toxic effect of mepivacaine on tumor cells was related to the mutation of oncogenes and oncogenes. The literature [20] clearly stated that the proliferation and metastasis of BCC are influenced by many factors. The literature [21] further claimed that mepivacaine greatly enhanced the release of inflammatory factors in BCC, promoted the phosphorylation of STAT3, and effectively decreased the release of anti-inflammatory factors. The literature [22] clarified that catecholamines stimulate the inflammatory response of the body and exert physiological effects such as stress restraint by affecting the release of inflammatory factors. This study also elucidated that elevated miR-27a in BCC can effectively inhibit the excessive release of inflammatory factors in mepivacaine-stimulated tumor cells, and it was hypothesized that miR-27a inhibits the toxic effects of mepivacaine on tumor cells by affecting the release of inflammatory factors. The literature [23] claimed that immune checkpoint inhibitors can lead to the release of multiple inflammatory factors in HCC and further stimulate tumor cell apoptosis. Thus, the lethal effect of immune response leading to tumor is almost related to the occurrence of inflammatory response.

IRE1, an important sensor on the endoplasmic reticulum membrane, is an important inducible protein for maintaining endoplasmic reticulum homeostasis. TRAF2, a key protein for transmitting apoptotic signals from the endoplasmic reticulum to the cytoplasm, can effectively inhibit the apoptotic process mediated by death receptors, and accordingly, the activated intracellular IRE1 protein can integrate with the downstream target protein TRAF2 to form a complex that inhibits apoptosis of tumor cells. This study clarified that mepivacaine effectively promoted the elevation of the apoptosis-related protein cleaved-caspase-3 and the decrease of Bcl-2/Bax in BCC. Elevated miR-27a in BCC effectively decreased cleaved-caspase-3 and enhanced Bcl-2/Bax. Mepivacaine had no effect on the activation of IRE1-TRAF2 signaling pathway, developing a close relationship between the mechanisms generating BCC apoptosis and the stimulation of intracellular inflammation. However, the protective effect of miR-27a on BCC should be related to the activation of the IRE1-TRAF2 signaling pathway.

The literature [24] indicated that IRE1 is in a free state after separation from endoplasmic reticulum molecular chaperones and undergoes oligomerization and dimerization, which then activates the IRE1 signaling pathway and elevates the downstream target protein TRAF2. The literature [25] suggested that IRE1 is a key protein that inhibits the apoptotic signaling pathway in tumor cells. Therefore, elevation of IRE1 could effectively reduce apoptotic proteins.

In brief, this project tested by in vitro experiments clarified that elevated miR-27a in BCC line MCF-7 was effective in reducing the toxic effects of mepivacaine on cells and enhancing cell progression. This mechanism is thought to be related to the activation of the IRE1-TRAF2 signaling pathway in BCC. These results may provide a theoretical basis for targeted treatment of BC in clinical practice.

## Figures and Tables

**Figure 1:** Detection of miR-27a in the cells of each group is via qPCR. Note:  ^*∗∗*^*P* < 0.01 versus the blank control.

**Figure 2:** Effect of miR-27a on the proliferation of BCC MCF-7. Note:  ^*∗∗*^*P* < 0.01 compared to control and ^##^*P* < 0.01 compared to mepivacaine.

**Figure 3:** Apoptosis of each group. Note: scale bar = 50 *μ*m,  ^*∗∗*^*P* < 0.01 compared with control, ^##^*P* < 0.01 compared with mepivacaine.

**Figure 4:** Cell migration capacity. Note:  ^*∗∗*^*P* < 0.01 versus control, ^##^*P* < 0.01 versus mepivacaine.

**Figure 5:** Levels of inflammatory factors in the cells. Note:  ^*∗∗*^*P* < 0.01 versus control, ^##^*P* < 0.01 versus mepivacaine.

**Figure 6:** Proteins associated with apoptosis in cells. Note:  ^*∗∗*^*P* < 0.01 versus control, ^##^*P* < 0.01 versus mepivacaine.

**Table 1:** PCR primers.

	The primer sequence
miR-27a	Forward: 5ʹ-GGTGTACACTGTAGCTAGTACGA-3ʹ
	Reverse: 5ʹ-TGATCGATAGCTAGTAAGTCAGGA-3ʹ

GAPDH	Forward: 5ʹ-GATCGTAGTCGATAAGCTAGAT-3ʹ
	Reverse: 5ʹ-ATAGCTAGCTAGCGATATCTAGCT-3ʹ

## Data Availability

The figures and tables used to support the findings of this study are included in the article.

## References

[1] Thorat M. A., Balasubramanian R. (2020). Breast cancer prevention in high-risk women. *Best Practice & Research Clinical Obstetrics & Gynaecology*.

[2] Lee A., Moon B.-I., Kim T. H. (2020). *BRCA1/BRCA2* pathogenic variant breast cancer: treatment and prevention strategies. *Annals of Laboratory Medicine*.

[3] Yu Y., Du H., Wei S. (2018). Adipocyte-derived exosomal MiR-27a induces insulin resistance in skeletal muscle through repression of PPAR*γ*. *Theranostics*.

[4] Tripathi A., Volsko C., Garcia J. P. (2019). Oligodendrocyte intrinsic miR-27a controls myelination and remyelination. *Cell Reports*.

[5] Jiang G., Shi W., Fang H., Zhang X. (2018). miR-27a promotes human breast cancer cell migration by inducing EMT in a FBXW7-dependent manner. *Molecular Medicine Reports*.

[6] Liu Y., Sun L., Ma Y., Wei B., Gao M., Shang L. (2019). High glucose and bupivacaine-induced cytotoxicity is mediated by enhanced apoptosis and impaired autophagy via the PERK-ATF4-CHOP and IRE1-TRAF2 signaling pathways. *Molecular Medicine Reports*.

[7] Zhang K., Liu H., Song Z. (2020). The UPR transducer IRE1 promotes breast cancer malignancy by degrading tumor suppressor microRNAs. *iScience*.

[8] Vieira W. A., Paranhos L. R., Cericato G. O., Franco A., Ribeiro M. A. G. (2018). Is mepivacaine as effective as lidocaine during inferior alveolar nerve blocks in patients with symptomatic irreversible pulpitis? A systematic review and meta-analysis. *International Endodontic Journal*.

[9] Cardoso J. M., Sá M., Reis H. (2018). Type II Quadratus Lumborum block for a sub-total gastrectomy in a septic patient. *Brazilian Journal of Anesthesiology (English Edition)*.

[10] Uematsu T., Nakashima K., Kikuchi M. (2020). The Japanese Breast Cancer Society clinical practice guidelines for breast cancer screening and diagnosis, 2018 edition. *Breast Cancer*.

[11] Hoerdemann M., Smith R. L., Hosgood G. (2017). Duration of action of mepivacaine and lidocaine in equine palmar digital perineural blocks in an experimental lameness model. *Veterinary Surgery*.

[12] Jordana M., Martens A., Duchateau L. (2016). Diffusion of mepivacaine to adjacent synovial structures after intrasynovial analgesia of the digital flexor tendon sheath. *Equine Veterinary Journal*.

[13] Visconti R. P., Tortamano I. P., Buscariolo I. A. (2016). Comparison of the anesthetic efficacy of mepivacaine and lidocaine in patients with irreversible pulpitis: a double-blind randomized clinical trial. *Journal of Endodontics*.

[14] Wang Y., Wang D., Jin Z. (2019). miR-27a suppresses TLR4-induced renal ischemia-reperfusion injury. *Molecular Medicine Reports*.

[15] Wang D., Si S., Wang Q. (2018). MiR-27a promotes hemin-induced erythroid differentiation of K562 cells by targeting CDC25B. *Cellular Physiology and Biochemistry*.

[16] Li W., Yu Z.-X., Ma B.-F. (2018). The increase of miR-27a affects the role of cisplatin on proliferation and migration capacities of liver cancer cells. *European Review for Medical and Pharmacological Sciences*.

[17] Adler D. M. T., Cornett C., Damborg P., Verwilghen D. R. (2016). The stability and microbial contamination of bupivacaine, lidocaine and mepivacaine used for lameness diagnostics in horses. *The Veterinary Journal*.

[18] Marrazzo E., Frusone F., Milana F. (2020). Mucinous breast cancer: a narrative review of the literature and a retrospective tertiary single-centre analysis. *The Breast*.

[19] Tofoli G. R., Cereda C. M. S., Groppo F. C. (2011). Efficacy of liposome-encapsulated mepivacaine for infiltrative anesthesia in volunteers. *Journal of Liposome Research*.

[20] Wu S., Li J., Ma T. (2021). MiR-27a regulates WNT3A and KITLG expression in cashmere goats with different coat colors. *Animal Biotechnology*.

[21] Zhu X., Zhang J., Sun H. (2014). Ubiquitination of inositol-requiring enzyme 1 (IRE1) by the E3 ligase CHIP mediates the IRE1/TRAF2/JNK pathway. *Journal of Biological Chemistry*.

[22] Zhang C., Kawauchi J., Adachi M. T. (2001). Activation of JNK and transcriptional repressor ATF3/LRF1 through the IRE1/TRAF2 pathway is implicated in human vascular endothelial cell death by homocysteine. *Biochemical and Biophysical Research Communications*.

[23] Zheng Q.-Y., Li P.-P., Jin F.-S. (2013). Ursolic acid induces ER stress response to activate ASK1–JNK signaling and induce apoptosis in human bladder cancer T24 cells. *Cellular Signalling*.

[24] Urano F., Wang X., Bertolotti A. (2000). Coupling of stress in the ER to activation of JNK protein kinases by transmembrane protein kinase IRE1. *Science*.

[25] Chen Y., Brandizzi F. (2013). IRE1: ER stress sensor and cell fate executor. *Trends in Cell Biology*.

